The article "Successful implementation of an enhanced recovery after surgery (ERAS) protocol reduces nausea and vomiting after infratentorial craniotomy for tumour resection: a randomized controlled trial" was retracted in 2020. Reasons: unreliable data; lack of ethics approval or compliance; concerns about the data.

# Successful implementation of an enhanced recovery after surgery (ERAS) protocol reduces nausea and vomiting after infratentorial craniotomy for tumour resection: a randomized controlled trial

**DOI:** 10.1186/s12883-020-01699-z

**Published:** 2020-04-22

**Authors:** Dan Lu, Yuan Wang, Tianzhi Zhao, Bolin Liu, Lin Ye, Lanfu Zhao, Binfang Zhao, Mingjuan Li, Lin Ma, Zhengmin Li, Jiangtao Niu, Wenhai Lv, Yufu Zhang, Tao Zheng, Yafei Xue, Lei Chen, Long Chen, Xude Sun, Guodong Gao, Bo Chen, Shiming He

**Affiliations:** 1 Department of Neurosurgery, Xi’an International Medical Center, Xi’an, China; 2 Department of Neurosurgery, Tangdu Hospital, The Fourth Military Medical University, Xi’an, China; 3 Department of Neurosurgery, Shaanxi Provincial People’s Hospital, Xi’an, China; 4 Department of Anesthesiology, Tangdu Hospital, The Fourth Military Medical University, Xi’an, China; 5 Department of Nutrition, Tangdu Hospital, The Fourth Military Medical University, Xi’an, China

**Keywords:** Enhanced recovery after surgery (ERAS), Postoperative nausea and vomiting (PONV), Infratentorial craniotomy, Anxiety, Sleep quality

## Abstract

**Background:**

Infratentorial craniotomy patients have a high incidence of postoperative nausea and vomiting (PONV). Enhanced Recovery After Surgery (ERAS) protocols have been shown in multiple surgical disciplines to improve outcomes, including reduced PONV. However, very few studies have described the application of ERAS to infratentorial craniotomy. The aim of this study was to examine whether our ERAS protocol for infratentorial craniotomy could improve PONV.

**Methods:**

We implemented an evidence-based, multimodal ERAS protocol for patients undergoing infratentorial craniotomy. A total of 105 patients who underwent infratentorial craniotomy were randomized into either the ERAS group (*n* = 50) or the control group (*n* = 55). Primary outcomes were the incidence of vomiting, nausea score, and use of rescue antiemetic during the first 72 h after surgery. Secondary outcomes included postoperative anxiety level, sleep quality, and complications.

**Results:**

Over the entire 72 h post-craniotomy observation period, the cumulative incidence of vomiting was significantly lower in the ERAS group than in the control group. Meanwhile, the incidence of vomiting was significantly lower in the ERAS group on postoperative days (PODs) 2 and 3. Notably, the proportion of patients with mild nausea (VAS 0–4) was higher in the ERAS group as compared to the control group on PODs 2 or 3. Additionally, the postoperative anxiety level and quality of sleep were significantly better in the ERAS group.

**Conclusion:**

Successful implementation of our ERAS protocol in infratentorial craniotomy patients could attenuate postoperative anxiety, improve sleep quality, and reduce the incidence of PONV, without increasing the rate of postoperative complications.

The article "Successful implementation of an enhanced recovery after surgery (ERAS) protocol reduces nausea and vomiting after infratentorial craniotomy for tumour resection: a randomized controlled trial" was retracted in 2020. Reasons: unreliable data; lack of ethics approval or compliance; concerns about the data.

**Trial registration:**

ChiCTR-INR-16009662, 27 Oct 2016, Clinical study on the development and efficacy evaluation of Enhanced Recovery After Surgery (ERAS) in Neurosurgery.

## Background

Neurosurgical patients are generally considered to have high risk of postoperative nausea and vomiting (PONV) according to the consensus guidelines for managing PONV [1]. Moreover, the incidence of PONV is more frequent after infratentorial procedures than supratentorial procedures [2]. Postoperative vomiting is not only unpleasant, but may also cause serious complications in neurosurgical patients, such as dehydration, electrolyte disturbances, aspiration and alkalosis. Poor control of PONV is associated with worse quality of life outcomes in the postoperative period, and is one of the most common reasons for prolonged hospitalization, which can contribute to healthcare costs.

Previous reports indicated that significant improvements in postoperative recovery can be achieved by implementing a standardized protocol of evidence-based treatments over the entire perioperative period [3, 4]. This concept of enhanced recovery after surgery (ERAS) was originally conceptualized by Kehlet to improve functional outcomes after surgery and decrease perioperative morbidity [5, 6]. ERAS protocols have been widely utilized in the perioperative period in several surgical fields such as colorectal surgery, urological surgery, and orthopedic surgery [7–9]. However, to the best of our knowledge, application of an ERAS protocol for infratentorial craniotomy has not yet been reported. Hagan et al. proposed some key components of ERAS applicable to craniotomy based on evidence available from other surgical specialties [10].

Based on this preliminary protocol and our own institutional experience, we presented a novel ERAS protocol for patients undergoing craniotomy at Tangdu hospital (Supplementary file). The aim of the present study was to prospectively evaluate whether this ERAS protocol significantly improved PONV after infratentorial craniotomy.

## Methods

### Study criteria

The present study was performed at Tangdu Hospital, which is affiliated with the Fourth Military Medical University. This study was approved by the institutional human research and ethics committee of Tangdu Hospital. This randomized control trial (RCT) was registered at the Chinese Trial Registry (**ChiCTR-INR-16009662**). In June 2016, we created a multidisciplinary committee, the ERAS Working Group, comprising of participants from neurosurgery, anesthesiology, in-patient and operative nursing, as well as nutrition services departments. All patients were given a complete explanation of the study protocol, drug, and numerical visual analogue scale (VAS) scores during the preoperational evaluation.

The article "Successful implementation of an enhanced recovery after surgery (ERAS) protocol reduces nausea and vomiting after infratentorial craniotomy for tumour resection: a randomized controlled trial" was retracted in 2020. Reasons: unreliable data; lack of ethics approval or compliance; concerns about the data.

After obtaining written and informed consent, 109 adult patients (American Society of anesthesiologists [ASA] physical status I or II, aged 17–75 years) undergoing infratentorial craniotomy between Oct 2016 and March 2018 were enrolled for this study. This study adopted a complete randomized grouping design. Before induction of anesthesia, the nurses responsible for patient allocation randomized the patients using a computer-generated random number table (Microsoft Excel 2013). Patients meeting the inclusion criteria were randomized using opaque sequentially numbered sealed envelopes into two groups: the control group and the ERAS group. Patients who got odd numbers were assigned to the control group, while those who got even numbers were assigned to the ERAS group. Exclusion criteria were intracranial trauma, microvacular decompression, pathology requiring emergency surgery, preoperative disturbance of consciousness, and presence of a confounding condition (e.g., pregnancy) or disease that could potentially impact postoperative recovery (e.g., paralysis, spinal deformity, autoimmune diseases, myocardial infarction, severe infection, liver and renal malfunction, or severe psychological or mental illness).

### ERAS protocol and conventional care

This prospective study was conducted to compare postoperative nausea, vomiting, anxiety and sleep quality in patients undergoing infratentorial craniotomy following the implementation of either an ERAS protocol or conventional care. The routine perioperative care of the control group was decided by individual surgeons and anesthetists, based on routine postoperative protocols (Supplementary file). The perioperative care of the ERAS group was managed according to the novel neurosurgical ERAS protocol described in this study. This ERAS protocol was developed based on an extensive review of the recent literature investigating evidenced-based perioperative care interventions and successful ERAS programs used in other operations [10]. Our novel ERAS protocol provided a standardized pathway that guided the perioperative management of patients undergoing craniotomy at Tangdu Hospital.

Briefly, the ERAS protocol consists of three main sections: Preoperatively, patients were evaluated and intervened based on the ERAS program that included preoperative counseling, preoperative functional status evaluation, preoperative smoking and alcohol abstinence (at least 2 weeks prior to surgery), mental state assessment, evaluation and prophylactic anti-thrombotic therapy, PONV risk score assessment, preoperative intestinal intervention (Glycerine Enema induction was given for patients with long history of constipation or ≥ 2 days without defecation.), nutritional assessment (NRS2002, nutritional status assessment, and PG-SGA were applied for nutritional assessment), and preoperative oral carbohydrate loading. During surgery, guidelines for the conduct of surgical and anesthetic management were implemented, including micro-invasive surgery for craniotomy, scalp incision anesthesia, non-opioid analgesia, absorbable skin suture, hypothermia avoidance, and fluid balance. Postoperatively, the pathway provided specific instructions for pain and PONV control, ambulation, urinary drainage, deep vein thrombosis (DVT) prophylaxis, oral intake, etc.

The article "Successful implementation of an enhanced recovery after surgery (ERAS) protocol reduces nausea and vomiting after infratentorial craniotomy for tumour resection: a randomized controlled trial" was retracted in 2020. Reasons: unreliable data; lack of ethics approval or compliance; concerns about the data.

PONV management is a vital component of our ERAS protocol. Preoperative PONV Simple Risk Assessment Scale was used to anticipate the relative risks of each individual. In the ERAS group, the high-risk patients (score ≥ 3) were administered tropisetron (a 5-HT_3_ antagonist, 2 mg) shortly before extubation for prophylaxis of postoperative vomiting. The patients in the control group did not receive prophylactic tropisetron. Postoperatively, the nausea VAS was used as one of the indications for PONV prevention and treatment in the ERAS group. After the patient was fully conscious, had stable vital signs, was extubated and breathing spontaneously, and could carry out basic commands, all ERAS patients were postoperatively monitored for PONV for 72 h. For patients who had moderate and severe nausea (VAS ≥ 5), tropisetron (2–5 mg, daily) was the first drug of choice. If tropisetron was ineffective, the combination of tropisetron (2–5 mg) and dexamethasone (5 mg), or the combination of tropisetron (2–5 mg) and droperidol (0.625–1.25 mg) was given until the VAS was ≤5. In the control group, antiemetics were administered only for patients with vomiting.

In addition, perioperative nutrition management was one of our foremost concerns. In the ERAS group, oral carbohydrate loading (i.e., maltodextrin fructose solution, 400 ml) was applied 2 h prior to the surgery. Postoperatively, oral water intake was permitted 4 h after surgery, while a polymeric nutritional supplement drink was given 8 h after surgery as tolerated by the patient in the ERAS group. In the control group, patients were allowed to take flow food on the postoperative day (POD) 1–2, semi-liquid food on POD 3–4, and solid food on POD 4–5. Thus, patients in the ERAS group had a shorter duration to first water intake (median 4 h in ERAS group vs. 10 h in control group), and first oral solid food intake (median 24 h vs. 96 h). Optimization of pain management was also a key element of our ERAS protocol. Local anesthetic administration with ropivacaine (0.2%) prior to scalp incision was applied as per our ERAS protocol. Scalp incision closure was achieved by absorbable intradermal running suturing in all ERAS patients. Postoperative morphine and equivalent opioids were not routinely prescribed in our patients of both group given their limited efficacy and wide range of side effects, unless a patient’s pain VAS score was greater than 7. Instead, nonopioid analgesia strategies such as the administration of intravenous acetaminophen or nonsteroidal antiinflammatory drugs (NSAIDs) were applied according to the intensity of the patient’s postoperative VAS score. Postoperatively, we applied same analgesia strategies to both groups patients. Early mobilization and shortened urinary catheterization were encouraged in our ERAS protocol. For deep vein thrombosis (DVT) evaluation and prophylaxis, patients in both groups were encouraged to perform frequent active and passive movement of their lower limbs. Mechanical DVT prophylaxis, which includes compressive stockings and intermittent pneumatic compression pump treatment, was uniformly performed for both groups after surgery. Additionally, many other ERAS elements are not specifically mentioned here. Supplementary file lists all the ERAS elements in detail.

The article "Successful implementation of an enhanced recovery after surgery (ERAS) protocol reduces nausea and vomiting after infratentorial craniotomy for tumour resection: a randomized controlled trial" was retracted in 2020. Reasons: unreliable data; lack of ethics approval or compliance; concerns about the data.

### Outcome measurements

This study was an observer-blinded RCT. Only those who collected and assessed outcomes were blinded. Various parameters were perioperatively assessed by blinded nurses. The same surgical and anesthesia teams performed all procedures. Anesthesia and monitoring were standardized for all patients. At our center, intravenous-inhalation combined anesthesia was adopted for craniotomy patients according to the anesthetist’s preference. Atropine and dexamethasone were preoperatively administrated to reduce gland secretion and minimize stress response. Propofol, sufentanil and rocuronium were used for anesthesia induction, while propofol, fentanyl and sevoflurane were used for anesthesia maintenance.

After the operation, all patients were postoperatively observed for 72 h. Vomiting was recorded as either present or absent by direct observation. The time and number of vomiting episodes were recorded. Both vomiting and retching were considered as emetic events. Nausea was scored using a 10-point VAS, with 0 indicating no nausea and 10 indicating the most severe nausea. Upon arrival in the intensive care unit, the patients were asked by the nurse to rate their nausea experience on the VAS device. This process was repeated every 8 h within 72 h in the surgical ward. While the patient was asleep, nausea was not assessed. Nausea was defined as a subjectively unpleasant sensation associated with the awareness of the urge to vomit; vomiting was defined as labored, spasmodic, rhythmic contraction of the respiratory muscles with or without expulsion of gastric contents from the mouth [11, 12]. Complete response was regarded as no vomiting or very mild nausea (VAS 0–2). All drugs given for PONV relief were documented.

The article "Successful implementation of an enhanced recovery after surgery (ERAS) protocol reduces nausea and vomiting after infratentorial craniotomy for tumour resection: a randomized controlled trial" was retracted in 2020. Reasons: unreliable data; lack of ethics approval or compliance; concerns about the data.

Subjectively rated anxiety was assessed on a 0 to 10 VAS (0 = very calm; 10 = very anxious). This parameter was postoperatively evaluated every morning. Subjectively rated quality of sleep, on a 0 to 10 VAS (0 = unable to sleep because of anxiety, 10 = deep and satisfactory sleep), was also postoperatively assessed immediately every morning. All postoperative surgical complications were judged and recorded by the investigator.

### Statistical analysis

The analyses were performed using SPSS (Ver. 19, IBM Corp., Armonk, NY). In neurosurgical patients, a 40% incidence of PONV after craniotomy was reported [13]. Based on the hypothesis that our ERAS protocol was expected to reduce the postoperative cumulative incidence of vomiting by at least 20%, a sample size of at least 41 patients per arm was calculated to have a power of 80% and a significance of 5%. To compensate for potential dropouts, 132 patients were enrolled. Interim analysis was planned when the minimal number of the predefined sample size was met.

The cumulative incidence of vomiting for 72 h after surgery was compared between the two groups using the Cox proportional hazards model. Other categorical variables were analyzed using the Fisher’s exact test and Chi-squared test, while continuous variables were analyzed using the t-test. Analysis of the parameters whose values were in large ranges was verified using the Mann-Whitney U-test. Continuous variables were expressed as the mean ± standard deviation; categorical variables were summarized as counts and percentage. A *p* value < 0.05 was deemed to indicate statistical significance.

## Results

### Demographics

A total of 132 patients from our hospital were enrolled in the present study. After exclusion, a total of 105 patients (55 in the control group and 50 in the ERAS group) were included in the analysis **(**Fig. 1**)**. There were no statistically significant differences in age, gender distribution, ASA class, and concomitant diseases between the two groups (Table 1). The relevant details of surgery and tumor pathology are summarized in Table 2. There were no significant differences in primary variables for surgery between the two groups. All patients woke up immediately after the interruption of anesthetics, and were fully conscious.

The article "Successful implementation of an enhanced recovery after surgery (ERAS) protocol reduces nausea and vomiting after infratentorial craniotomy for tumour resection: a randomized controlled trial" was retracted in 2020. Reasons: unreliable data; lack of ethics approval or compliance; concerns about the data.

**Fig. 1:** Flow diagram of CONSORT study design

**Table 1:** Patient demographics

Parameter	Control group (*n* = 55)	ERAS group (*n* = 50)	*P* value
Mean age, years	48.7 ± 12.5	47.0 ± 13.0	0.51
Gender			
Male, n(%)	20 (36%)	21 (42%)	0.68
Female, n(%)	35 (64%)	29 (58%)	
Mean BMI, kg/m2	23.0 ± 2.7	23.3 ± 2.9	0.55
ASA classification			
ASA I, n(%)	18 (33%)	19 (38%)	0.57
ASA II, n(%)	37 (67%)	31 (62%)	
Concomitant diseases			
Cardiac/hypertension, n(%)	8 (15%)	10 (20%)	0.61
Smoker, n(%)	10 (18%)	12 (24%)	0.48
Liver/gall bladder, n(%)	1 (2%)	3 (6%)	0.35
Lung, n(%)	3 (5%)	5 (1%)	0.47
Diabetes mellitus, n(%)	11 (20%)	7 (14%)	0.45
Miscellaneous, n(%)	7 (13%)	5 (10%)	0.76

Data are expressed as mean ± SD or number of patients (%). P value indicates the comparison between control group and ERAS group. ASA, American Society Anesthesiologists

**Table 2:** Surgery characteristics

Parameter	Control group (n = 55)	ERAS group (n = 50)	*P* value
Infratentorial approach			
CPA meningioma, n(%)	10 (18%)	9 (18%)	0.64
Acoustic neuroma, n(%)	10 (18%)	12 (24%)	
Trigeminal neuroma, n(%)	4 (7%)	3 (6%)	
Glioma, n(%)	17 (31%)	15 (30%)	
Hemangioblastoma, n(%)	6 (11%)	5 (10%)	
CPA cholesteatoma, n(%)	8 (15%)	6 (12%)	
Tumor size, cm	3.1 ± 1.0	2.9 ± 1.0	0.30
Mean duration of surgery, minutes	322.9 ± 125.5	308.2 ± 110.4	0.52
Blood loss > 300 ml, n(%)	15 (27%)	10 (20%)	0.49
Blood transfusion, n(%)	7 (13%)	5 (10%)	0.76
Use of colloid, n(%)	20 (36%)	19 (38%)	1.00

Data are expressed as mean ± SD or number of patients (%). *P* value indicates the comparison between control group and ERAS group. CPA, cerebellopontine angle

### PONV and the use of antiemetics

The two primary goals of this study were to assess the PONV and antiemetics consumption (Table 3). The preoperative PONV risk assessment was performed on all patients of the two groups. Twenty (40%) patients in the ERAS group were high-risk individuals of PONV versus 18 (33%) patients in the control group (*p* = 0.54). Based on the preoperative PONV risk score, the high-risk patients in the ERAS group received PONV prophylaxis (40%, RR: 74.61, 95% CI: 4.35–1278, *p* < 0.0001). The cumulative incidence of vomiting over the 72 h post-craniotomy observation period was significantly lower in the ERAS group patients than in the control group patients (Cox proportional test; HR: 0.47, 95% CI: 0.23–0.96, *p = 0.03) (Fig. 2).

**Table 3:** Postoperative nausea and vomiting outcomes

Phase	Parameter	Control group (n = 55)	ERAS group (n = 50)	P value
Pre-operation	PONV simple risk assessment, n(%)	55 (100%)	50 (100%)	–
	High-risk individuals, n(%)	18 (33%)	20 (40%)	0.54
Post-operation	PONV prophylaxis, n(%)	0 (0%)	20 (40%)	< 0.01
	Complete response			
	POD 1, n(%)	22 (40%)	23 (46%)	0.56
	POD 2, n(%)	22 (40%)	31 (62%)	0.03
	POD 3, n(%)	29 (53%)	37 (74%)	0.02
	Vomiting			
	POD 1, n(%)	15 (27%)	9 (18%)	0.35
	POD 2, n(%)	12 (22%)	3 (6%)	0.02
	POD 3, n(%)	8 (15%)	1 (2%)	0.03
	Nausea score (VAS), POD 1			0.33
	Mild (0–4), n(%)	24 (44%)	29 (58%)	
	Moderate (5–6), n(%)	16 (29%)	11 (22%)	
	Severe (7–10), n(%)	15 (27%)	10 (20%)	
	Nausea score (VAS), POD 2			0.01
	Mild (0–4), n(%)	25 (45%)	35 (70%)	
	Moderate (5–6), n(%)	16 (29%)	11 (22%)	
	Severe (7–10), n(%)	14 (25%)	4 (8%)	
	Nausea score (VAS), POD 3			0.02
	Mild (0–4), n(%)	33 (60%)	40 (80%)	
	Moderate (5–6), n(%)	13 (24%)	9 (18%)	
	Severe (7–10), n(%)	9 (16%)	1 (2%)	
	Antiemetic medication administration			
	POD 1			
	All antiemetics, no. of requests	15 (27%)	21 (42%)	0.14
	tropisetron, mean mg/user	2.8 ± 1.2	3.0 ± 1.1	0.61
	POD 2			
	All antiemetics, no. of requests	12 (22%)	15 (30%)	0.50
	tropisetron, mean mg/user	2.5 ± 0.8	2.7 ± 1.0	0.63
	POD 3			
	All antiemetics, no. of requests	8 (15%)	10 (20%)	0.60
	tropisetron, mean mg/user	2.3 ± 0.5	2.4 ± 0.7	0.60

Data are expressed as number of patients (%). P value indicates the comparison between control group and ERAS group. POD, Postoperative day; PONV, postoperative nausea and vomiting; VAS, Visual Analogue Scale

The article "Successful implementation of an enhanced recovery after surgery (ERAS) protocol reduces nausea and vomiting after infratentorial craniotomy for tumour resection: a randomized controlled trial" was retracted in 2020. Reasons: unreliable data; lack of ethics approval or compliance; concerns about the data.

**Fig. 2:** The cumulative incidence of vomiting in patients of the ERAS group and the control group. The cumulative incidence of vomiting over the 72 h post-craniotomy observation period was significantly lower in the ERAS group patients than in the control group patients. Cumulative incidence was calculated by the number of new cases during a period divided by the number of subjects at risk in the population

There was no difference in the rate of complete response between the two groups on POD 1 (*p* = 0.56). However, the rates of complete response were significantly higher in the ERAS group on PODs 2 and 3 (POD 2: 31/50, 62% in ERAS vs. 22/55, 40% in control; RR: 2.44, 95% CI: 1.11–5.37, *p* = 0.03. POD 3: 37/50, 74% in ERAS vs. 29/55, 53% in control; RR: 2.55, 95% CI: 1.11–5.82, *p* = 0.02). Meanwhile, the incidence of vomiting was significantly lower in the ERAS group on PODs 2 and 3 (POD 2: 3/50, 6% in ERAS vs. 12/55, 22% in control; RR: 0.22, 95% CI: 0.06–0.86, *p* = 0.02. POD 3: 1/50, 2% in ERAS vs. 8/55, 15% in control; RR: 0.11, 95% CI: 0.01–0.99, p = 0.03).

Additionally, more patients in the ERAS group scored their nausea as mild level on POD 1 as compared to the control group, but the difference was not significant (*p* = 0.33). Notably, on PODs 2 or 3, the nausea score revealed a significantly higher proportion of mild nausea in the ERAS group as compared to the control group (POD 2: 35/50, 70% in ERAS vs. 25/55, 45% in control; RR: 2.80, 95% CI: 1.25–6.26, *p* = 0.01. POD 3: 40/50, 80% in ERAS vs. 33/55, 60% in control; RR: 2.66, 95% CI: 1.10–6.41, *p* = 0.03).

The article "Successful implementation of an enhanced recovery after surgery (ERAS) protocol reduces nausea and vomiting after infratentorial craniotomy for tumour resection: a randomized controlled trial" was retracted in 2020. Reasons: unreliable data; lack of ethics approval or compliance; concerns about the data.

Lastly, antiemetics were not more frequently used in the ERAS group than in the control group on the POD 1 (*p* = 0.14). In addition, on PODs 2 and 3, there were no significant differences between the two groups, although the nausea score and the vomiting incidence were lower in the ERAS group. Postoperatively, tropisetron, which was regarded as the first-line antiemetic, was given when a patient complained of moderate or serious nausea or if vomiting occurred. The total amount of tropisetron doses per user in each group were almost identical on PODs 1, 2 and 3 (POD 1: *p* = 0.61; POD 2: *p* = 0.63; POD 3: *p* = 0.60).

### Postoperative anxiety and sleep quality

The two secondary goals of this study were to assess the postoperative anxiety level and the associated sleep disturbances (Table 4). During PODs 0 to 3, the ERAS group patients had a self-rated anxiety level that was significantly lower than that of the control group patients (POD 1: *p* = 0.01; POD 2: *p* < 0.01; POD 3: p = 0.01). The quality of sleep on PODs 1, 2 and 3 was rated significantly better by the ERAS group patients (i.e., a higher VAS score) than the controls (POD 1: *p* = 0.02; POD 2: *p* = 0.03; POD 3: p = 0.03).

**Table 4:** Immediate postoperative anxiety level and sleep quality

Parameter	Control group (n = 55)	ERAS group (n = 50)	*P* value
Anxiety level, mean VAS score			
POD 1	6.5 ± 1.9	5.6 ± 1.7	0.01
POD 2	5.7 ± 2.0	4.8 ± 1.7	< 0.01
POD 3	3.9 ± 1.7	3.1 ± 1.4	0.01
Sleep quality, mean VAS score			
POD 1	6.5 ± 1.3	7.2 ± 1.5	0.02
POD 2	5.4 ± 1.2	5.9 ± 1.3	0.03
POD 3	4.0 ± 1.3	4.5 ± 1.3	0.03

Data are expressed as mean ± SD. P value indicates the comparison between control group and ERAS group. POD, Postoperative day; VAS, Visual Analogue Scale

### Postoperative complications

The characteristics of the surgical complications were similar in the two groups (Table 5). In the present study, there were no serious postoperative complications, such as related death or disturbance of consciousness. One ERAS group patient and two control group patients suffered intracranial hemorrhage, but none of them required reoperation. Neurological deficits occurred in 7 patients from the ERAS group and 11 patients from the control group. Of these patients, most of them were diagnosed to be facial paralysis secondary to acoustic neuroma surgery. All patients were conservatively treated with medication for their complications. Three patients in the ERAS group and two patients in the control group had surgical site infections, and recovered after sterile dressing change and antibiotic treatment. One patient in the control group had an intracranial infection, and recovered after antibiotic treatment and lumbar drainage.

The article "Successful implementation of an enhanced recovery after surgery (ERAS) protocol reduces nausea and vomiting after infratentorial craniotomy for tumour resection: a randomized controlled trial" was retracted in 2020. Reasons: unreliable data; lack of ethics approval or compliance; concerns about the data.

**Table 5:** Postoperative complications

Parameter	Control group (n = 55)	ERAS group (*n* = 50)	P value
Mortality, n(%)	0 (0%)	0 (0%)	–
Disturbance of consciousness, n(%)	0 (0%)	0 (0%)	–
Intracranial infection, n(%)	1 (2%)	0 (0%)	1.00
Hemorrhage*, n(%)	2 (4%)	1 (2%)	1.00
Cerebral infarction, n(%)	0 (0%)	0 (0%)	–
Neuro deficits**, n(%)	11 (20%)	7 (14%)	0.44
Aspiration, n(%)	0 (0%)	0 (0%)	–
Surgical site infection/ subcutaneous effusion, n(%)	2 (4%)	3 (6%)	0.66

Data are expressed as number of patients (%). P value indicates the comparison between control group and ERAS group. * Hemorrhage refers to small amount of epidural hematoma or surgical area hemorrhage, not including intracranial hemorrhage which needs re-operation. ** Neuro deficits refers to cranial-nerve palsies after operation, including facial paralysis, ophthalmoplegia, trigeminal nerve injury, etc.

### Multivariable associations

Univariate analysis showed significant association between a lower incidence of vomiting on POD 2 and the following parameters in all patients of the two groups: male, low-risk individuals of PONV, preoperative mouth-rinsing, duration of surgery < 315 min, did not use colloid, and PONV prophylaxis. Multivariate logistic regression model, including variables with *p* < 0.20 in the univariate analysis, was used to evaluate independent predictors of vomiting on POD 2. The multivariable model is shown in Table 6. High-risk individuals of PONV (RR: 170.609, 95% CI: 5.773–5042.077, *p* = 0.003), duration of surgery > 315 min (RR: 22.611, 95% CI: 1.307–391.205, *p* = 0.032), and use of colloid (RR: 44.161, 95% CI: 2.754–708.126, *p* = 0.007) were significant risk factors for vomiting on POD 2. Preoperative mouth-rinsing (RR: 0.007, 95% CI: 0.000–0.331, *p* = 0.012), and PONV prophylaxis (RR: 0.012, 95% CI: 0.000–0.479, *p* = 0.019) were independent predictors for a lower incidence of vomiting on POD 2 in the multivariate analysis.

**Table 6:** Multivariate logistic regression for predictors of postoperative vomiting on POD 2 in all patients

Variable	RR (95% CI)	P value
Gender	8.930 (0.957–83.347)	0.055
High-risk individuals of PONV	170.609 (5.773–5042.077)	0.003
Preoperative mouth-rinsing	0.007 (0.000–0.331)	0.012
Duration of surgery > 315 min	22.611 (1.307–391.205)	0.032
Use of colloid	44.161 (2.754–708.126)	0.007
PONV prophylaxis	0.012 (0.000–0.479)	0.019

Abbreviations: POD: Postoperative day

The article "Successful implementation of an enhanced recovery after surgery (ERAS) protocol reduces nausea and vomiting after infratentorial craniotomy for tumour resection: a randomized controlled trial" was retracted in 2020. Reasons: unreliable data; lack of ethics approval or compliance; concerns about the data.

## Discussion

The development of a novel, multidisciplinary, evidence-based, neurosurgical ERAS protocol for elective craniotomy was associated with shortened postoperative hospital length of stay and rapid recovery after surgery [14]. We also investigated whether the ERAS protocol was superior to conventional perioperative management in infratentorial craniotomy patients. This was the first randomized, controlled trial to demonstrate that the ERAS protocol for elective infratentorial craniotomy was associated with a significantly lower cumulative incidence of postoperative vomiting, nausea and anxiety, and better postoperative quality of sleep, which led to an accelerated functional recovery. Additionally, the surgical complications were not significantly different between the ERAS and control groups.

PONV is usually defined as any nausea or vomiting occurring within the first 24–72 h after surgery. Protracted PONV can be extremely distressing to patients and is one of the most common causes of dehydration, acid-base disturbances, and electrolyte imbalance after surgery [15]. The physical act of vomiting may raise intracranial or cerebral intravascular pressure, jeopardizing cerebral perfusion and hemostasis. However, there is a lack of uniform standards in the definitions of “nausea” and “vomiting”. In some studies, analysis of PONV is restricted to vomiting, whereas in others, nausea and vomiting are recorded together. Nausea is a subjective sensation requiring activation of neural pathways, which eventually project to areas of the cerebral hemispheres dealing with conscious sensations [16]. Nausea is not always followed by vomiting. In some studies, nausea and vomiting were considered as two different biological phenomena [17], and were separately analyzed. In neurosurgical patients, a 40–80% incidence of PONV within 24 h after craniotomy was reported [18, 19]. Moreover, several observational studies demonstrated that infratentorial surgeries were associated with a higher incidence of PONV [2, 20, 21]. For instance, Meng concluded that PONV frequently occurs in adults recovering from retromastoid craniectomy with microvascular decompression of cranial nerves [22]. A possible biological reason for this may be because the surgical area is close to the area postrema (vomiting center) [23]. It receives input from the chemoreceptor trigger zone, vestibular apparatus, cerebellum, and solitary tract nucleus [24]. Inadvertent or unavoidable interference with these areas may cause release of humoral factors that may be stimuli for PONV [2]. Conceivably, infratentorial craniotomy was an especially high-risk factor for PONV in patients undergoing craniotomy.

The article "Successful implementation of an enhanced recovery after surgery (ERAS) protocol reduces nausea and vomiting after infratentorial craniotomy for tumour resection: a randomized controlled trial" was retracted in 2020. Reasons: unreliable data; lack of ethics approval or compliance; concerns about the data.

Our ERAS protocol incorporated recent evidences and expert opinions for effective perioperative PONV management. In our ERAS protocol, preoperative PONV Simple Risk Assessment Scale was applied to anticipate the relative risk of each patient, and associated prophylaxis was given based on the result [25]. In a systematic review, the factors considered to have a potential effect on the risk of experiencing PONV included female gender, a history of motion sickness or PONV, nonsmoking status, and use of postoperative opioids [25]. The incidence of PONV with the presence of 0, 1, 2, 3, or all 4 of these risk factors were 10, 20, 40, 60, and 80%, respectively [26]. All patients who had the PONV risk > 40% according to the simplified risk score were evaluated as high-risk populations. In the ERAS group, these high-risk patients were administered tropisetron shortly before extubation for prophylaxis of postoperative vomiting. At present, there is no evidence of any difference in efficacy and harm of different 5-HT_3_ receptor antagonists (tropisetron, ondansetron, granisetron, and dolasetron). Therefore, for the treatment of PONV symptoms, we use the cheapest 5-HT_3_ receptor antagonist (tropisetron) in our hospital pharmacy. 5-HT_3_ receptor antagonists were proven to be effective for the prevention of postoperative emesis after craniotomy, with minimal adverse effects [27–29]. They do not produce sedation, extrapyramidal reactions or drug interactions with other anesthetic drugs. However, when anti-nausea and anti-vomiting efficacies were separately analyzed, 5-HT_3_ receptor antagonist was found to have a greater anti-vomiting effect than an anti-nausea effect [30]. In contrast, there is more anti-nausea and less anti-vomiting efficacy with the dopamine receptor antagonist (droperidol) [31]. Therefore, there is evidence of an increased antiemetic efficacy with a combination of droperidol and 5-HT_3_ receptor antagonist in the surgical setting [32]. However, in a recent warning by the Food and Drug Administration (FDA), droperidol, when used in antiemetic doses, was associated with prolongation of QTc interval and fatal arrhythmias [23]. The FDA recommended that droperidol should not be used as a first-line therapy. Besides, similar effectiveness was observed when a 5-HT_3_ receptor antagonist was combined with droperidol or dexamethasone [33].

Based on the above, in our ERAS protocol, the intervention measures (nausea score, VAS ≥ 5) were applied for attenuating symptoms according to nausea score after surgery. We tracked both antiemetics use and patients’ reporting of nausea. The results showed that more patients in the ERAS group reported mild nausea and complete response (VAS 0–4) on PODs 2 and 3 than in control group (Table 3). The results of this study also showed that our PONV management in the ERAS protocol was associated with a lower cumulative incidence of vomiting after surgery as compared to the conventional care. Although more ERAS patients requested antiemetics in comparison with the control patients on POD 1, there was no statistically significant difference in postoperative tropisetron consumption per user between the two groups. These phenomena could be explained by the efficacy of our PONV management strategy. Based on the use of nausea VAS, more postoperative patients in the ERAS group who needed antiemetics treatment were selected. Our PONV management strategy in the ERAS protocol was effective for preventing PONV on PODs 2 and 3, without any increase in tropisetron dosage per user.

The article "Successful implementation of an enhanced recovery after surgery (ERAS) protocol reduces nausea and vomiting after infratentorial craniotomy for tumour resection: a randomized controlled trial" was retracted in 2020. Reasons: unreliable data; lack of ethics approval or compliance; concerns about the data.

Our ERAS protocol for elective craniotomy focussed on enhanced recovery and shorter hospital stay after surgery [14]. It is well known that craniotomy can substantially disturb the homeostasis of the body and cause extensive surgical stress [34]. Hence, an adequate stress response is advantageous. However, excessive stress can lead to a pathological state. An excessive stress response may predispose the patient to an increased risk of cardiovascular and cerebrovascular complications, nutrient malabsorption, and delayed convalescence. Our ERAS strategies, including prophylaxis and management of PONV, DVT, preoperative fasting, incisional local anesthesia, wound closure (Dural, subcutaneous tissue and skin are sutured by absorbable suture), urinary catheter duration, and surgical site pain, are aimed to reduce the stress-related responses in patients after surgery. Less stress response may lead to less inflammation and pain, with subsequently less postoperative vomiting [35, 36]. Scalp nerve block have been showed to reduce VAS pain scores and analgesics requirements after surgery. It is possible that the lower incidence of PONV in the ERAS group was related to less intraoperative remifentanil consumption and postoperative analgesics use. This may be another reason for improving PONV [37]. In addition, multivariate analysis revealed that preoperative mouth-rinsing (Compound Chlorhexidine Gargle) and PONV prophylaxis were independent predictors for a lower incidence of vomiting on POD 2 in all patients **(**Table 6**)**. These predictors may be interpreted as the determinants for reducing vomiting on POD 2 in the ERAS group.

There is mounting evidence to suggest that pain and anxiety may also increase the incidence of PONV after surgery [38, 39]. Our ERAS strategies incorporated recent evidence and expert opinions in designing the analgesic protocols [40, 41]. Our previous study showed a significant improvement in pain control after surgery with ERAS implementation [14]. In addition, patients in the ERAS group were able to achieve earlier oral water/food intake, ambulation, and removal of the urinary catheter after surgery. These ERAS strategies could reduce postoperative discomfort and anxiety, and improve sleep quality in patients with infratentorial craniotomy (Table 4). The ERAS patients showed improved mental state. Therefore, it is not surprising that the ERAS patients in this study had a lower incidence of PONV when compared to the control group.

The article "Successful implementation of an enhanced recovery after surgery (ERAS) protocol reduces nausea and vomiting after infratentorial craniotomy for tumour resection: a randomized controlled trial" was retracted in 2020. Reasons: unreliable data; lack of ethics approval or compliance; concerns about the data.

There were no differences in the incidence of postoperative complications between the ERAS and control groups in this study (Table 5). Limited by the case number, these results might not reflect the positive influences of the ERAS protocol in this aspect. However, this study demonstrated the efficacy of the ERAS protocol, without an increased complication risk.

This study had some limitations. First, due to the need for active participation of the patients, this trial could not be blinded in the clinical setting. Blinding of the patients’ study arm was employed in this study for those who collected data and assessed outcomes. Second, this study reported data concerning a relatively small number of patients who underwent infratentorial craniotomy. Therefore, further evaluation of the protocol in larger population is warranted in the future.

## Conclusion

Implementation of our ERAS pathway for infratentorial craniotomy was associated with a reduction in postoperative nausea and vomiting, without any increase in the rate of postoperative complications. Future studies are needed to identify the individual interventions that contribute the most to quality of recovery in the acute postoperative period, as well as the long-term effects of ERAS implementation on chronic postoperative PONV and antiemetic use.

## Supplementary information

**Additional file 1:.**

## Data Availability

All data generated or analysed during this study are included in this published article.

## Abbreviations

PONV: postoperative nausea and vomiting
ERAS: Enhanced Recovery After Surgery
RCT: randomized control trial
VAS: visual analogue scale
ASA: american society of anesthesiologists
DVT: deep vein thrombosis
PODs: postoperative days
CPA: cerebellopontine angle
